The article "NOSH-NBP, a Novel Nitric Oxide and Hydrogen Sulfide- Releasing Hybrid, Attenuates Ischemic Stroke-Induced Neuroinflammatory Injury by Modulating Microglia Polarization" was retracted in 2023. Reasons: duplicated images; original data or images not available; unreliable data; unreliable results or conclusions.

# NOSH-NBP, a Novel Nitric Oxide and Hydrogen Sulfide- Releasing Hybrid, Attenuates Ischemic Stroke-Induced Neuroinflammatory Injury by Modulating Microglia Polarization

**DOI:** 10.3389/fncel.2017.00154

**Published:** 2017-05-26

**Authors:** Jing Ji, Pengjun Xiang, Tingting Li, Li Lan, Xiaole Xu, Guo Lu, Hui Ji, Yihua Zhang, Yunman Li

**Affiliations:** ^1^State Key Laboratory of Natural Medicines, Department of Pharmacology, China Pharmaceutical UniversityNanjing, China; ^2^State Key Laboratory of Natural Medicines, Department of Physiology, China Pharmaceutical UniversityNanjing, China; ^3^School of Pharmacy, Nantong UniversityNantong, China; ^4^State Key Laboratory of Natural Medicines, Center of Drug Discovery, China Pharmaceutical UniversityNanjing, China

**Keywords:** NOSH-NBP, ischemic stroke, neurovascular unit, microglial/macrophage polarization, TLR4/MyD88/NF-κB pathway, NLRP3 inflammasome, PPARγ

## Abstract

NOSH-NBP, a novel nitric oxide (NO) and hydrogen sulfide (H_2_S)-releasing hybrid, protects brain from ischemic stroke. This study mainly aimed to investigate the therapeutic effect of NOSH-NBP on ischemic stroke and the underlying mechanisms. *In vivo*, transient middle cerebral artery occlusion (tMCAO) was performed in C57BL/6 mice, with NO-NBP and H_2_S-NBP as controls. NO and H_2_S scavengers, carboxy-PTIO and BSS, respectively, were used to quench NO and H_2_S of NOSH-NBP. *In vitro*, BV_2_ microglia/BMDM were induced to the M1/2 phenotype, and conditioned medium (CM) experiments in BV_2_ microglia, neurons and b.End3 cerebral microvascular endothelial cells (ECs) were performed. Microglial/macrophage activation/polarization was assessed by flow cytometry, Western blot, RT-qPCR, and ELISA. Neuronal and EC survival was measured by TUNEL, flow cytometry, MTT and LDH assays. Transmission electron microscopy, EB extravasation, brain water content, TEER measurement and Western blot were used to detect blood–brain barrier (BBB) integrity and function. Interestingly, NOSH-NBP significantly reduced cerebral infarct volume and ameliorated neurological deficit, with superior effects compared with NO-NBP and/or H_2_S-NBP in mice after tMCAO. Both NO and H_2_S-releasing groups contributed to protection by NOSH-NBP. Additionally, NOSH-NBP decreased neuronal death and attenuated BBB dysfunction in tMCAO-treated mice. Furthermore, NOSH-NBP promoted microglia/macrophage switch from an inflammatory M1 phenotype to the protective M2 phenotype *in vivo* and *in vitro*. Moreover, the TLR4/MyD88/NF-κB pathway and NLRP3 inflammasome were involved in the inhibitory effects of NOSH-NBP on M1 polarization, while peroxisome proliferator activated receptor gamma signaling contributed to NOSH-NBP induced M2 polarization. These findings indicated that NOSH-NBP is a potential therapeutic agent that preferentially promotes microglial/macrophage M1–M2 switch in ischemic stroke.

## Introduction

Ischemic stroke, one of the primary causes of disability and death worldwide, contributes for up to 85% of total stroke incidence (Liu et al., 2015; Jian et al., 2016). Fundamental approaches to acute stroke therapy are blood flow recovery and neuroprotection. Currently, intravenous thrombolysis initiated within 3 h of stroke onset is the only approved and validated therapy for acute ischemic stroke, and is used in a very small percentage of patients at most centers (Denorme et al., 2016). Meanwhile, cerebral ischemia reperfusion injury is a severe complication of thrombolysis therapy, which limits its clinical application for ischemic stroke.

It is widely acknowledged that therapeutic interventions for ischemic stroke should not only prevent neuronal death, but also target multiple brain cell types in an attempt to protect their structural and functional integrity as well as normal interactions (del Zoppo, 2006). The NVU is comprised of neurons, glial cells and BBB, in which cell–cell interactions underlie the basis for normal brain function (Stanimirovic and Friedman, 2012). On the contrary, signaling dysfunction in the NVU results in disease. Hence, to be successful, stroke therapy should be broadly effective in each component of the NVU. Additionally, the important crosstalk between neurons, glial cells, and BBB becomes more prominent in the penumbral region, a functionally impaired but not dead area of the ischemic brain, which is pathophysiologically characterized by hypoxia/reoxygenation stress, BBB disruption, edema, and active inflammation (da Fonseca et al., 2014).

As an important component of the NVU, microglia are the major immune cells in the brain, building the first line of defense against brain injury (Elali and Rivest, 2013). However, they play a dual role in ischemic stroke injury. Indeed, in response to specific stimulations, microglia alter their phenotypes and functions, after classical (M1) or alternative (M2) activation (Kobayashi et al., 2013). M1-polarized microglia are characterized by the production and release of proinflammatory mediators. In contrast, M2-polarized microglia reduce inflammation and possess neuroprotective properties (Xia et al., 2015). It was confirmed *in vitro* that M1 microglia exacerbate neuronal damage, whereas M2 counterparts prevent neuronal death after ischemia (Hu et al., 2012; Girard et al., 2013). In turn, ischemia-induced neurons drive the microglial M2-M1 switch by releasing soluble factors and/or shedding cell components (Shu et al., 2016). As the core NVU component, the BBB is a gatekeeper for maintaining the fragile homeostasis of the central nervous system (CNS), and its disruption is a key event in the pathogenesis of ischemic stroke, which contributes to intracerebral vasogenic edema and hemorrhagic transformation (Fan et al., 2014; Cheon et al., 2016). When ischemia occurs in the brain, microglia produce cytokines and chemokines, and stimulate adhesion on ECs, potentiating damage to BBB viability and integrity (Yenari et al., 2006). In particular, classical microglial activation by LPS impairs the BBB function by regulating important molecules involved in BBB integrity, such as occludin and ZO-1 (Sumi et al., 2010). Although the above findings suggest that microglia participate in EC damage and BBB disruption, the effects of different microglia polarization phenotypes on the BBB function in ischemia stroke remain uncharacterized.

Nitric oxide and H_2_S are important gasotransmitters in the brain. As the first known gasotransmitter, NO has both cytoprotective and cytotoxic effects. Apart from cytotoxic effects of peroxynitrite formation with superoxide anion, NO exerts its cytoprotective effects partly by acting as a key modulator of immune and inflammatory responses. For instance, NO inhibits NF-κB activation, which is a frequent target of immunosuppressive and anti-inflammatory molecules (Hattori et al., 2004). Furthermore, NO suppresses NLRP3 inflammasome activation, which is a multi-protein complex that triggers the maturation of the pro-inflammatory cytokines IL-1β and IL-18 (Mao et al., 2013; Mishra et al., 2013). Additionally, compounds containing NO-donor moieties possess increased anti-inflammatory properties (Hauss et al., 1999; Hauss-Wegrzyniak et al., 1999; Wenk et al., 2000, 2002). As the newest gasotransmitter, H_2_S is traditionally considered a poisonous gas and environmental pollutant. Evidence accumulated over the last decade reveals the potential value of H_2_S in the treatment of CNS diseases, including stroke and neurodegenerative diseases (Kida and Ichinose, 2015; Cui et al., 2016). Exogenous H_2_S donors confer neuroprotection in ischemic stroke, at least in part, owing to their anti-inflammatory properties (Yin et al., 2013). Moreover, some NO and H_2_S-releasing compounds (NOSH-compounds) exhibit enhancive anti-inflammatory effects (Kodela et al., 2013; Nia et al., 2013). Lee et al. (2013) reported that a NO and H_2_S-releasing compound, NOSH-ASA, has significant anti-inflammatory properties in the CNS.

Previous reports demonstrated that NO or H_2_S-donor derivatives of NBP, NO-NBP (zjm-289), and H_2_S-NBP (8e) exhibit anti-thrombosis, anti-platelet aggregation and neuroprotective properties (Zhuang et al., 2010; Wang X. et al., 2014). NBP was approved by the State Food and Drug Administration (SFDA) of China as a new anti-ischemic drug for stroke in 2002. With beneficial effects on stroke, NBP, however, has limited clinical application due to insufficient efficacy. Many attempts on the structural modification of NBP have been carried out to yield an ideal anti-ischemic stroke drug. Since both NO and H_2_S may have a crucial role in ischemic stroke, we recently synthesized NOSH-NBP (8d), a novel NBP derivative, that could release both of these gasotransmitters (Yin et al., 2016). NOSH-NBP was shown to possess a more potent activity than NBP in cerebral ischemia reperfusion injury with preventive administration, including anti-platelet aggregation, anti-oxidant activity, and alleviation on infract volume and edema. Considering its potential effect, further exploration and research is necessary for NOSH-NBP in ischemic stroke. However, the therapeutic potential of NOSH-NBP on cerebral ischemia reperfusion injury, and the underlying mechanisms remain unknown.

Hence, this study aimed: (1) to investigate the therapeutic effect of NOSH-NBP on cerebral ischemia reperfusion injury; (2) to compare NOSH-NBP, NO-NBP, and H_2_S-NBP for their activities in cerebral ischemia reperfusion injury; (3) to determine the underlying mechanism of NOSH-NBP against cerebral ischemia reperfusion injury; (4) to provide further information for future development of NO and H_2_S-donating drugs.

## Materials and Methods

### Chemicals

NOSH-NBP (purity > 99%), NO-NBP (purity > 99%), and H_2_S-NBP (purity > 99%) were synthesized by the Center of Drug Discovery, China Pharmaceutical University. Their molecular structures are shown in **Figure 1**. Carboxy-PTIO (PTIO, a reported NO scavenger) and BSS (a known H_2_S scavenger) were supplied from Shenzhen Simeiquan Biotechnology, Co., Ltd ADTOH (purity > 99.9%) and 4-HBN (purity > 99%) were purchased from Shanghai Boyle Chemical, Co., Ltd. These compounds were dissolved in normal saline.

**FIGURE 1:** **Structural components of NO-NBP (A)**, H_2_S – NBP **(B)**, and NOSH-NBP **(C).** The parent compound, NBP is shown in the shaded boxes. ADTOH released H_2_S and ONO_2_ released NO, both shown in dotted ellipses (*j* = 4; *k* = 6; *m* = 2; *n* = 5).

### Animal Care

E16-18 embryos from pregnant female and male counterparts (6–8 weeks old, 20–23 g) were provided by Comparative Medicine Centre of Yangzhou University (Yangzhou, China). All animal protocols (NO: 14311010053, 05/22/2016) were approved by China Pharmaceutical University in accordance with the guidelines of the National Institutes of Health throughout the study.

### Establishment of an Ischemia and Reperfusion (I/R) Model

Transient middle cerebral artery occlusion was considered ischemia/reperfusion injury, and performed as described previously (Cheon et al., 2016). In brief, following right common carotid artery (CCA), internal carotid artery (ICA) and external carotid artery (ECA) exposure, a monofilament (BeiJing Sunbio Biotech, China) with a round tip was inserted into the ICA through the ECA stump and gently pushed toward the MCA. The regional cerebral blood flow (rCBF) in the MCA field was monitored by Iaser Doppler flowmetry (LDF 100C; BIOPAC Systems, Goleta, CA, United States). After occlusion for 1 h, the monofilament was immediately withdrawn to allow reperfusion for 3 days. The core body temperature was maintained at 37.0 ± 0.5°C by a temperature-controlled heating pad (CMA 190; Carnegie Medicin, Sweden) during the whole procedure. Mice with unsuccessful MCAO (rCBF falling by less than 75%) and failed reperfusion (rCBF raised to less than 70% of baseline) were excluded.

### Experimental Protocol

To determine the therapeutic effects of test compounds on ischemic stroke and the underlying mechanisms, 285 mice were randomly divided into nine groups, i.e., sham (sham operation), model (tMCAO + vehicle), tMCAO + NO-NBP (0.4 mm/kg), tMCAO + H_2_S-NBP (0.4 mm/kg), tMCAO + PTIO + NOSH-NBP (0.4 mm/kg), tMCAO + BSS + NOSH-NBP (0.4 mm/kg), tMCAO + NOSH-NBP (0.4 mm/kg), tMCAO + NOSH-NBP (0.2 mm/kg) and tMCAO + NOSH-NBP (0.1 mm/kg) groups. Vehicle and drugs were orally administered immediately at the beginning of reperfusion, once every 24 h.

### Infarct Volume Assessment

Three days after reperfusion, mice were sacrificed and brains were sliced into five coronal sections from the frontal tip. They were stained with 2% of TTC (Sigma, United States) for 20 min at 37°C and fixed in 10% formalin at 4°C overnight. The infarct tissues remained unstained, while viable tissues were stained deep red based on the normal mitochondrial function. The border of the infarct zone was outlined with an image processing software. The infarct volume rate was calculated and expressed as a percentage of total brain volume, as described previously (Jian et al., 2016).

### Assessment of Neurological Deficits

At 24, 48, and 72 h of reperfusion, neurological deficits in the animals were blindly evaluated by the Longa’s method (Longa et al., 1989) with minor modifications. According to the different degrees of motor deficits, neurological deficit scores were classified into a five-point scale: 0, no neurological deficit; 1, flexion to contralateral torso and forepaw; 2, circling to the left side but normal posture at rest; 3, leaning to the contralateral side at rest; 4, no spontaneous motor activity and lost consciousness.

### Immunofluorescence for MAP2 Detection and Terminal Deoxy-Ribonucleotide Transferase dUTP Nick end Labeling (TUNEL) Staining

Three days after reperfusion, the animals were perfused with cold saline to remove the blood. Brain specimens were quickly removed and fixed in 4% paraformaldehyde for 24 h, and immersed in 30% sucrose in PBS for 48 h, for staining as described previously (Mlinar et al., 2016). Brain sections (frozen) were cut at a thickness of 5 μm on a cryostat vibratome (VT 2800 N; Leica, Germany). Frozen sections were fixed in acetone for 20 min at -20°C, and endogenous peroxidase was inhibited by 1% H_2_O_2_ methanol for 20 min at room temperature (25°C). Subsequently, sections were blocked with 5% goat serum (Sigma-Aldrich, United States) at room temperature for 2 h, and incubated with a primary antibody against MAP2 (1: 200 in PBS) (Cell Signaling Technology, United States) overnight at 4°C. The next day, brain sections were incubated in the dark with fluorescently labeled secondary antibodies for 2 h at room temperature (25°C) following three washes in PBS. Then, brain sections were stained by the TUNEL assay kit (Roche, Switzerland) according to the manufacturer’s instructions and counterstained with DAPI for 5 min at room temperature (25°C). The samples were analyzed by laser scanning microscopy.

### Transmission Electron Microscopy

Three days after reperfusion, the mice were perfused with cold normal saline through the left ventricle to remove blood from the vessels. The penumbral region from the brain tissues was fixed with 3% glutaraldehyde buffered in 0.1 M sodium cacodylate (pH 7.2). After 3-days of storage, each sample was rinsed in PBS and fixed in cacodylate-buffered 1% osmium tetroxide. Subsequently, post-fixed samples were dehydrated in graded ethanol and embedded in PolyBed 812 to obtain ultra-thin (90 nm) sections using a microtome. The sections were stained with 3% lead citrate, and subsequently assessed on a transmission electron microscope (JEOL, JEM-2000EX, Japan).

### Evans Blue (EB) Extravasation

Evans blue extravasation was used to assess BBB integrity, as described previously (Jie et al., 2015). Briefly, animals were administered with EB (2% in saline, 4 mg/kg) by via the tail vein injection after 3 days of reperfusion. At 2 h after EB injection, the mice were perfused with saline through the left ventricle under anesthesia. Following harvest, brain specimens were divided into left (contralateral) and right (ipsilateral) hemispheres. Then, the hemispheres were homogenized and centrifuged. Supernatants were collected and analyzed at 620 nm on a spectrometer. EB leakage of each hemisphere was quantified by a standard curve, and expressed as μg per gram of wet weight.

### Brain Water Content Measurement

Blood–brain barrier integrity impairment can also be reflected by brain water content. Three days after reperfusion, brain samples were immediately removed and weighed (wet weight) after sacrifice, for brain water content measurement as described previously. Dry weight was measured after samples were dried at 105°C for 1 day. Brain water content was then derived as [(wet weight-dry weight)/wet weight] × 100%.

### Flow Cytometry Analysis of CD11b Expression

Ischemic hemisphere samples obtained from each group after 3 days of reperfusion were dissociated with 800 U DNase I and 2 mg/ml papain in hank’s balanced salt solution (HBSS) at 37°C for 60 min. After filtration with 70 μm cell strainers (Becton Dickinson, United States) to generate a single cell suspensions, immune cells were separated by centrifugation using 20% Percoll in PBS at 5000 rpm for 10 min. Microglia/macrophages were enriched using CD11b affinity beads (Miltenyi Biotec, United States) and incubated in blocking solution (anti-CD16/32 antibody; BD Biosciences, United States). Then, the cells were stained with PE-Cy7-CD11b fluorescently labeled antibody at 4°C for 30 min and assessed by flow cytometry (Becton Dickinson, San Diego, CA, United States). Data analysis was performed with the CellQuest software (BD Bioscience, United States).

### Cell Culture and *In Vitro* Experiments

BV_2_ microglia and b.End3 cerebral microvascular endothelial cells (ECs) were obtained from Shanghai Institute of Cell Bank (Shanghai, China), and cultured in DMEM containing 10% fetal bovine serum (FBS, Gibco, United States) in a humidified atmosphere with 5% CO_2_. For primary macrophage culture, bone marrow-derived macrophages (BMDMs) were flushed from C57BL/6 male mice (6–8 weeks old, 20–23 g) femurs and incubated for 7 days with a medium containing GM-CSF. Culture of primary neurons was performed as described previously with some modifications. Briefly, brain samples were obtained from E16-18 embryos of pregnant C57BL/6 mice. Subsequently, cortex samples were dissected and digested with 800 U DNase I and 2 mg/ml papain at 37°C for 40 min, and gently shaken every 5 min. Digestion was stopped with FBS, and cell suspensions were filtered with a strainer (40 μm; Millipore, United States). Following centrifugation for 5 min at 1000 rpm, the dissociated cells were resuspended in DMEM containing 10% FBS and plated onto poly-l-lysine-coated plates. After 4 h of incubation, the culture medium was replaced by the Neurobasal medium (Gibco, United States) supplemented with 2% B27 (Gibco, United States). The cortical neurons were maintained in primary culture medium for 7 days and used in subsequent experiments.

For M1 phenotype induction, microglia/macrophages were treated with LPS (Sigma, United States) (100 ng/mL) and IFN-γ (PeproTech, China) (20 ng/mL) for 24 h. For M2 phenotype induction, microglia/macrophages were treated with IL-4 (PeproTech, China) (20 ng/mL) for 24 h.

To achieve OGD, cells were placed in a humidified 37°C incubator, with a gas mixture of 94% N_2_ and 5% CO_2_ introduced for about 15 min to almost deplete O_2_ (<1%). The cell culture medium was replaced with d-glucose-free DMEM (Gibco, United States) for OGD.

We first determined whether ischemia and the test compounds affected M1/M2 polarization of microglia/macrophages. BV_2_ microglia/macrophages in 6-well plate (1 × 10^5^) were subjected to 3 h OGD. Then, non-OGD or post-OGD microglia/macrophages were treated with LPS+IFN-γ, IL-4, ADTOH, 4-HBN, NO-NBP, H_2_S-NBP, NOSH-NBP or a combination of these agents for 24 h. Afterward, the expression levels of M1 (CCL3, IL-1β, and TNF-α) and M2 (CD206, Ym1/2, and Arg1) markers were evaluated.

To evaluate the effect of the test compound-treated M1 microglial CM on post-OGD primary neuron survival, cell supernatants were collected from the M1 microglia, as well as NO-NBP, H_2_S-NBP, and NOSH-NBP-treated M1 counterparts. The primary neurons in 96-well plates (1 × 10^5^/well) or 6-well plates (1 × 10^6^/well) were treated with normal medium or CM from the above microglia after 60 min of OGD. Primary neurons were incubated with CM for 24 h, and neuron apoptosis, cell viability, and LDH release were assessed.

To determine the role of microglia polarization in BBB viability and integrity under hypoxic/ischemic conditions, and evaluate the effects of test compound-treated M1 microglial CM on post-OGD ECs survival, the CM was collected from M0 microglia, M1 microglia, M2 microglia, as well as NO-NBP, H_2_S-NBP, or NOSH-NBP-treated M1 microglia. ECs in 96-well plates (1 × 10^4^/well) or transwell inserts (0.5 × 10^4^/cm^2^) were treated with normal or CM from the above microglia after 3 h of OGD. The ECs were incubated with the CM for 24 h, and cell viability, LDH release, TEER, and occludin and ZO-1 levels were assessed.

To investigate the regulatory mechanisms of NOSH-NBP on microglia polarization, BV2 microglia in 6-well plates (1 × 105/well) were treated with LPS+IFN-γ, IL-4, NOSH-NBP, TLR4 siRNA, GM9662 (PPARγ antagonist; Sigma, United States) or a combination of these agents for 24 h, and the related signaling pathway was explored.

### TLR4 Silencing

SiRNA transfection was used to down-regulate TLR4. Control siRNA and TLR4 siRNA (Abilene, United States) were transfected into BV_2_ microglia using Lipofectamine 2000 (Invitrogen, Carlsbad, CA, United States) for 24 h. The transfection efficiency of BV_2_ microglia was determined by Western blotting.

### Western Blotting

Total protein was extracted from the penumbral region of ischemic hemispheres, different conditions-treated ECs or BV_2_ microglia as described previously (Wang et al., 2016). Then, 20 μg of protein samples were subjected to 10–15% Bis-Tris gel electrophoresis and transferred onto a 0.2 μm polyvinylidene fluoride membranes (Millipore Corporation, United States). The membranes were blocked with 5% non-fat dry milk-TBS-0.1% Tween 20 for 2 h and washed. Then, the membranes were incubated with primary antibodies against TLR4, MyD88, p-p65, p65 (1:200, all from Santa Cruz, CA, United States), PPARγ, NLRP3, caspase-1, lba1, CD68 (1:1000, both from Abcam, United States), occludin, ZO-1 and β-actin (1:1000, all from Cell Signaling Technology, United States), overnight at 4°C. This was followed by incubation with appropriate horseradish conjugated secondary antibodies for 2 h. Immunoreactivity was detected by the BeyoECL Plus kit (Beyotime, China) on an image system (ChmiScope 2850; Clinx Science Instruments, China); band intensities were analyzed and calculated.

### RNA Extraction and Quantitative Real-Time Reverse Transcription-PCR

Total RNA was extracted from the penumbral region of ischemic hemisphere or BV_2_ microglia using the RNeasy Mini kit (QIAGEN, Netherlands). Then, cDNA was prepared from 2 μg of total RNA using a Transcriptor First Strand cDNA Synthesis kit (Roche Diagnostics, Germany). Quantitative real-time reverse transcription-PCR (RT-PCR) was perormed on M × 3000P (Agilent Technologies, United States) with synthetic primers and SYBR Green (Agilent Technologies, United States). Amplification was carried out for 45 cycles at 95°C for 10 s, 60°C for 10 s, and 72°C for 15 s, after holding at 50°C for 2 min and 95°C for 10 min. The specific primers are listed in **Table 1**. Relative expression levels were calculated using the 2-^[Ct experimental sample–Ct internal control sample (GAPDH)]^ method.

**Table 1:** The primer sequences using quantitative RT-PCR of M1 and M2 markers.

M1 marker (5′–3′)		M2 marker (5′-3′)	
CCL3	ATGCAAGTTCAGCTGCCTGC	CD206	CTTCGGGCCTTTGGAATA AT
	ATGCCGTGGATGAACTGAGG		TAGAAGAGCCCTTGGGTTGA
IL-1β	TGGAAAAGCGGTTTGTCTTC	Ym1/2	CAGGGTAATGAGTGGGTTGG
	TACCAGTTGGGGAACTCTGC		CACGGCACCTCCTAAATTGT
TNF-α	CATCTTCTCAAAATTCGAGTGAC	Arg1	GTGAAGAACCCACGGTCTGT
	TGGGAGTAGACAAGGTACAACCC		GCCAGAGATGCTTCCAACTG

### Flow Cytometry Analysis of Primary Neuron Apoptosis

Following the manufacturer’s instructions, apoptosis was assessed using FITC Annexin V apoptosis detection kit I (BD Biosciences, United States). Briefly, primary neurons were washed twice with cold PBS and resuspended in 100 μL binding buffer. Then, 5 μL FITC Annexin V and 5 μL PI were added to cells under gentle mixing and incubated for 15 min at room temperature in the dark. After addition of 400 μL binding buffer, the pre-incubated cells were detected by flow cytometry (Becton Dickinson, San Diego, CA, United States). The percentages of apoptotic to normal cells were assessed by the CellQuest software (BD Bioscience, United States).

### Cell Viability Assessment

After 24 h incubation of neurons or ECs with CM, cell deaths of OGD-neurons or OGD-ECs were measured by the MTT assay and LDH activity. 50 μl of the MTT solution (5 mg/ml; Sigma, United States) was added to each well for an additional 4 h. After careful removal of the medium, 190 μl DMSO was added to dissolve the dark blue formazan crystals. Finally, absorbance at 550 nm was read on a microplate reader (Bio-Rad Laboratories, Ltd, China). To confirm cell death, LDH activity was determined using a LDH kit (JianCheng Bioengineering Institute, China) according to the manufacturer’s instructions.

### Trans-endothelial Electrical Resistance (TEER) Measurement

Trans-endothelial electrical resistance, which reflects the permeability of TJs to sodium ions, was measured on a Millicell-ERS voltohmmeter (Millipore, United States). Three readings were taken per insert and averaged.

### Enzyme-Linked Immunosorbent Assay (ELISA) for IL-1β, IL-18, IL-6, and TNF-α Detection in Brains and Cell Culture Supernatants

Three days after reperfusion, infarcted half brains were collected and homogenized for ELISA analysis. After BV_2_ microglia being treated with different conditions, culture supernatants were collected for ELISA analysis. The concentrations of IL-1β, IL-18, IL-6, and TNF-α were detected by specific mouse ELISA kits (Biolegend, United States) according to the manufacturer’s instructions.

### Statistical Analysis

Data are mean ± standard deviation (SD), from at least three independent experiments. Data were analyzed by one way analysis of variance (ANOVA), with *post hoc* Tukey test (LSD procedure) applied to assess group pairs. *P <* 0.05 was considered statistically significant. Figures were generated with Statistical Analysis System (GraphPad Prism 5; GraphPad Software, Inc., San Diego, CA, United States).

## Results

### Effects of NO-NBP, H_2_S-NBP, and NOSH-NBP on Neurological Deficit Score and Infarct Volume in Response to tMCAO Injury

Neurological behavioral tests indicated that NO-NBP (0.4 mm/kg) and H_2_S-NBP (0.4 mm/kg) both attenuated neurological dysfunction caused by tMCAO injury. NOSH-NBP (0.4, 0.2, and 0.1 mm/kg) remarkably decreased the neurological deficit scores in a time- and dose-dependent manner. With extending treatment time, NOSH-NBP at 0.4 mm/kg was more potent than NO-NBP and/or H_2_S-NBP in decreasing the neurological deficit scores (**Figures 2A–C** and Supplementary Figure S2). Similarly, a significant and dose-dependent reduction of pale-colored region (infarct region) was observed in NOSH-NBP (0.4, 0.2, and 0.1 mm/kg) treated mice, by 47.26, 23.86, and 11.13%, respectively, compared with values of the model group. NO-NBP (0.4 mm/kg) and H_2_S-NBP (0.4 mm/kg) also decreased the infarct volume (23.29 and 25.4% respectively), but far less than NOSH-NBP (0.4 mm/kg) (*P* < 0.05). Furthermore, the effects of NO and H_2_S on the therapeutic ability of NOSH-NBP were investigated. Improving effects of NOSH-NBP on neurological dysfunction and infarct volume were lowered after treatment with carboxy-PTIO (a known NO scavenger) or bismuth (III) subsalicylate (BSS, a reported H_2_S scavenger) (**Figures 2D,E**). These data were sufficient to confirm that NOSH-NBP could serve as a feasible agent to lessen cerebral ischemia/reperfusion injury in this animal model.

**FIGURE 2:** **Effects of test compounds (NO-NBP, H_2_S-NBP, and NOSH-NBP) on neurological deficit scores and infarct volumes in tMCAO mice.** The model- group and test compounds- groups underwent tMCAO; the sham group underwent the same surgical procedure without the filament insertion. After MCAO completion, mice in test compounds groups were administered with NO-NBP (0.4 mm/kg), H_2_S-NBP (0.4 mm/kg), NOSH-NBP (0.4 mm/kg)+PTIO, NOSH-NBP (0.4 mm/kg)+BSS or NOSH-NBP (0.4, 0.2 and 0.1 mm/kg) for 3 days. **(A–C)** Neurological deficit evaluation was performed at 24, 48, and 72 h after reperfusion according to the Longa’s method with minor modifications. **(D)** Representative examples of TTC staining from each treatment group of mice. Infarct volume percentages data indicated in **(E)** were calculated as infarct area/whole area. The neurological deficit scores were present as mean (*n* = 18) and the infarct volume percentage were presented as mean ± SD (*n* = 6). Data were analyzed by one-way analysis of variance (ANOVA) followed by *post hoc* Tukey test: ^∗∗∗^*P <* 0.001, ^∗∗^*P <* 0.01, ^∗^*P <* 0.05.

### Effects of NO-NBP, H_2_S-NBP, and NOSH-NBP on Neuronal Apoptosis in Response to tMCAO Injury

To determine the neuroprotective effects of test compounds on cerebral ischemia, TUNEL assay was performed. Compared with the model group, markedly less TUNEL-positive cells in the penumbral area of tMCAO mice were observed after NOSH-NBP (0.4 mm/kg) treatment (*P* < 0.001). NO-NBP at 0.4 mm/kg and H_2_S-NBP at 0.4 mm/kg tended to restore tMCAO-induced increased amounts of TUNEL-positive cells, although no statistical difference was found. Treatment with NO-NBP, H_2_S-NBP, and NOSH-NBP also reduced the percentage of TUNEL-positive neurons (*P* < 0.05, *P* < 0.05, and *P* < 0.001, respectively). NOSH-NBP displayed better neuroprotective effects compared with NO-NBP and H_2_S-NBP (both *P* < 0.05; **Figures 3A–C**). NOSH-NBP treatment with carboxy-PTIO or BSS confirmed that lack of NO or H_2_S weakened the anti-neuronal apoptosis activity of NOSH-NBP, suggesting that NO and H_2_S both contributed to neuroprotection by NOSH-NBP.

**FIGURE 3:** **Effect of NO-NBP, H_2_S-NBP, and NOSH-NBP on neuronal apoptosis in the penumbral area of tMCAO mice.** The model- group and test compounds- groups underwent tMCAO; the sham group underwent the same surgical procedure without the filament insertion. After MCAO being performed, mice in test compounds group were administrated with NO-NBP (0.4 mm/kg), H_2_S-NBP (0.4 mm/kg), NOSH-NBP (0.4 mm/kg) + PTIO, NOSH-NBP (0.4 mm/kg) + BSS or NOSH-NBP (0.4, 0.2, and 0.1 mm/kg) for 3 days. **(A)** Representative photographs of TUNEL. These images were analyzed by Image Pro Plus, and each datum was presented as **(B)** TUNEL positive cells and **(C)** neurons in per mm^2^ within five random independent view fields. The data were presented as mean ± SD (*n* = 3) and were analyzed by one-way ANOVA followed by *post hoc* Tukey test: ^∗∗∗^*P* < 0.001, ^∗∗^*P* < 0.01, ^∗^*P* < 0.05.

### Effects of NO-NBP, H_2_S-NBP, and NOSH-NBP on BBB Integrity in Response to tMCAO Injury

The ultrastructural characteristics of cerebral microvessels were observed by transmission electron microscopy. Cerebro-microvessels of the sham group exhibited normal characteristics of ECs and basement membranes. Swollen mitochondria with vague crista and blurred membranes in ECs and edema in the basement membranes were detected in the tMCAO group, and restored to some extent by NO-NBP (0.4 mm/kg), H_2_S-NBP (0.4 mm/kg), and NOSH-NBP (0.4 mm/kg) (**Figure 4A**). EB leakage into the ischemic (ipsilateral) brain parenchyma and brain water content was further confirmed. In comparison with the model group, NOSH-NBP (0.4, 0.2, and 0.1 mm/kg) dose dependently alleviated EB extravasation and edema formation. NO-NBP (0.4 mm/kg) and H_2_S-NBP (0.4 mm/kg) inhibited EB leakage (*P* < 0.05, *P* < 0.01), but had no significant effects on brain water content (**Figures 4B,C**). Additionally, the levels of occludin and ZO-1, BBB function-associated proteins, were tremendously decreased by tMCAO injury. NOSH-NBP (0.4, 0.2, and 0.1 mm/kg) significantly increased occludin and ZO-1 levels in a dose-dependent manner (**Figures 4D,E**). Overall, NOSH-NBP at 0.4 mm/kg was more potent than NO-NBP or H_2_S-NBP alone in repairing BBB breakdown. However, NO- or H_2_S-elimination in NOSH-NBP both greatly decreased its protective effect on BBB by treatment with carboxy-PTIO or BSS.

**FIGURE 4:** **Effect of NO-NBP, H_2_S-NBP, and NOSH-NBP on BBB breakdown in tMCAO mice.** The model- group and test compounds- groups underwent tMCAO; the sham group underwent the same surgical procedure without the filament insertion. After MCAO completion, mice in test compound groups were administered with NO-NBP (0.4 mm/kg), H_2_S-NBP (0.4 mm/kg), NOSH-NBP (0.4 mm/kg)+PTIO, NOSH-NBP (0.4 mm/kg)+BSS or NOSH-NBP (0.4, 0.2, and 0.1 mm/kg) for 3 days. **(A)** Electron micrographs of microvessel cross sections of rats in the **(*a*)** control, **(*b*)** model, **(*c*)** tMCAO + NO-NBP (0.4 mm/kg), **(*d*)** tMCAO + H_2_S-NBP (0.4 mm/kg), **(*e*)** tMCAO + NO-NBP (0.4 mm/kg) + PTIO, **(*f*)** tMCAO + NO-NBP (0.4 mm/kg) + BSS and **(*g*)** tMCAO + NOSH-NBP (0.4 mm/kg) groups. BM, basement membrane; M, mitochondria; V, vacuolation. **(B)** Quantitative analysis of EB content in ischemic (ipsilateral) cortex and non-ischemic (contralateral) cortex (*n* = 4). **(C)** Quantitative analysis of brain water content in the brains (*n* = 6). **(D)** Representative Western blot membranes for occludin and ZO-1 proteins expressions. **(E)** Quantitative analysis of occludin and ZO-1 proteins expressions levels (*n* = 3). Data are expressed as the mean ± SD and were analyzed by one-way ANOVA followed by *post hoc* Tukey test: *^∗∗∗^P <* 0.001, *^∗∗^P* < 0.01, *^∗^P* < 0.05.

### Effects of NO-NBP, H_2_S-NBP, and NOSH-NBP on Microglia/Macrophage Activation and M1/M2 Polarization in Response to tMCAO Injury

Microglial/macrophage activation and deactivation in the ischemic brain were investigated by flow cytometry and Western blotting. As shown in **Figures 5A,B**, flow cytometry demonstrated that CD11b levels in individual microglia/macrophages were enhanced in tMCAO mice, and suppressed by NO-NBP (0.4 mm/kg), H_2_S-NBP (0.4 mm/kg), and NOSH-NBP (0.4, 0.2, and 0.1 mm/kg), to varying degrees. Similarly, Western blot demonstrated that the protein levels of lba1 and CD68 were increased in tMCAO mice, and suppressed by NO-NBP (0.4 mm/kg), H_2_S-NBP (0.4 mm/kg), and NOSH-NBP (0.4, 0.2, and 0.1 mm/kg) (**Figures 5C,D**).

**FIGURE 5:** **Effect of NO-NBP, H_2_S-NBP, and NOSH-NBP on microglia/macrophage activation and relative M1/M2 activation in ischemic brain.** The model- and test compound-groups underwent tMCAO while the sham group underwent the same surgical procedure without the filament insertion. After MCAO being performed, mice in test compound-groups were administered with NO-NBP (0.4 mm/kg), H_2_S-NBP (0.4 mm/kg), NOSH-NBP (0.4 mm/kg) + PTIO, NOSH-NBP (0.4 mm/kg) + BSS or NOSH-NBP (0.4, 0.2, and 0.1 mm/kg) for 3 days. **(A)** A representative profile of CD11b expression. **(B)** Quantitative analysis of the mean fluorescence intensity (MFI) of CD11b (*n* = 3). **(C)** Representative Western blot membranes for lba1 and CD68. **(D)** Quantitative analysis of lba1 and CD68 protein expression levels (*n* = 3). Quantitative analysis of mRNA expression of the M1 markers **(E)** CCL3, **(F)** IL-1β and **(G)** TNF-α (*n* = 6). Quantitative analysis of mRNA expression of the M2 markers **(H)** CD206, **(I)** Ym1/2, and **(J)** Arg1 (*n* = 6). Data were expressed as the mean ± SD and were analyzed by one-way ANOVA followed by *post hoc* Tukey test: *^∗∗∗^P <* 0.001, *^∗∗^P* < 0.01, *^∗^P* < 0.05.

As shown in **Figures 5E–J**, tMCAO injury both increased the mRNA levels of M1 (CCL3, IL-1β, and TNF-α) and M2 (CD206, Ym1/2, and Arg1) markers. NO-NBP (0.4 mm/kg), H_2_S-NBP (0.4 mm/kg), and NOSH-NBP (0.4, 0.2, and 0.1 mm/kg) inhibited the expression levels of M1 markers and conversely increased M2 marker levels. NOSH-NBP at 0.4 mm/kg was more effective in inhibiting microglial/macrophage activation and promoting M1–M2 switch compared with NO-NBP and H_2_S-NBP administered alone. Moreover, NO and H_2_S also contributed to these effects of NOSH-NBP, as reflected by carboxy-PTIO or BSS treatment. Interestingly, NO- or H_2_S-elimination in NOSH-NBP blunted its inhibitory effects on M1 polarization; however, different from M2 polarization, only H_2_S-elimination of NOSH-NBP alleviated the positive effects of NOSH-NBP on M2 polarization.

### Effects of ADTOH, 4-HBN, NO-NBP, H_2_S-NBP, and NOSH-NBP on M1/M2 Polarization in Response to OGD, LPS+IFN-γ, or IL-4

In addition to NO-NBP and H_2_S-NBP, ADTOH (a common H_2_S-releasing agent) and 4-HBN (a common NO-releasing agent) were used as control treatments. OGD injury mimicked ischemic stroke *in vitro*, and not only increased the expression levels of M1 markers (CCL3, IL-1β, and TNF-α) but also enhanced those of M2 markers (CD206, Ym1/2, and Arg1). Consistent with *in vivo* findings, NOSH-NBP significantly inhibited OGD-induced over-expression of M1 markers (CCL3, IL-1β, and TNF-α) and further increased the expression levels of M2 markers (CD206, Ym1/2, and Arg1). For specific microglial/macrophage M1 and M2 polarization induction, LPS+IFN-γ and IL-4 immensely enhanced the levels of M1 markers (CCL3, IL-1β, and TNF-α) and M2 markers (CD206, Ym1/2, and Arg1), respectively. NO-NBP, H_2_S-NBP, ADTOH, 4-HBN, and NOSH-NBP inhibited the over-expression of M1 markers (CCL3, IL-1β, and TNF-α) caused by LPS+IFN-γ (**Figures 6A–C** and Supplementary Figures S1A–C). NOSH-NBP was the most effective test reagent and 4-HBN the least potent. High expressions of M2 markers (CD206, Ym1/2, and Arg1) induced by IL-4 were further enhanced by NO-NBP, H_2_S-NBP, ADTOH and NOSH-NBP, but not 4-HBN (**Figures 6D–F** and Supplementary Figures S1D–F). Taken together, *in vitro* data demonstrated that NOSH-NBP promoted M1–M2 switch.

**FIGURE 6:** **Effect of ADTOH, 4-HBN, NO-NBP, H_2_S-NBP, and NOSH-NBP on microglial M1/M2 polarization *in vitro*.** BV_2_ microglia were treated with OGD, LPS (100 ng/mL) + IFN-γ (20 ng/mL), IL-4 (20 ng/mL), NO-NBP (10 μM), H_2_S-NBP (10 μM), ADTOH (10 μM), 4-HBN (10 μM), NOSH-NBP (10 μM) or a combination of these treatments. Quantitative analysis of mRNA expression levels of the M1 markers **(A)** CCL3, **(B)** IL-1β, and **(C)** TNF-α (*n* = 6). Quantitative analysis of mRNA expression levels of the M2 markers **(D)** CD206, **(E)** Ym1/2, and **(F)** Arg1 (*n* = 6). Data are expressed as the mean ± SD and were analyzed by one-way ANOVA followed by *post hoc* Tukey test: *^∗∗∗^P <* 0.001, *^∗∗^P* < 0.01, *^∗^P* < 0.05.

### Effects of M1 Microglial Conditioned Medium after NO-NBP, H_2_S-NBP, and NOSH-NBP-Treatment on Post-OGD Neuron Survival

To clarify the neuroprotective role of modulating microglia polarization, post-OGD primary neurons were incubated with samples of microglial CM for 24 h. As shown in **Figure 7**, M1 microglia CM exacerbated OGD-induced neuronal death, as revealed by increased neuronal apoptosis and LDH release, as well as reduced cell viability. In comparison with the M1 microglia CM group, CMs from NO-NBP, H_2_S-NBP, and NOSH-NBP-treated M1 microglia all attenuated OGD-induced neuronal damage by inhibiting neuronal apoptosis and LDH release, while promoting cell viability. In addition, NOSH-NBP was more potent in preventing post-OGD neurons from damage caused by M1 cells, which coincided with its effect on microglial polarization.

**FIGURE 7:** **Effect of NO-NBP, H_2_S-NBP, or NOSH-NBP-treated M1 microglial condition medium on post-OGD primary neuronal survival.** BV_2_ microglia were treated with LPS (100 ng/mL) + IFN-γ (20 ng/mL), NO-NBP (10 μM), H_2_S-NBP (10 μM), NOSH-NBP (10 μM) or a combination of these agents for 24 h, followed by the collection of conditioned media (CM). After 1 h OGD, primary neurons were incubated with different CM of microglia (M1 CM, NO-NBP M1 CM, H_2_S-NBP M1 CM, or NOSH-NBP M1 CM), respectively. **(A)** Photographs of mouse cortical neurons taken by phase-contrast microscopy: **(*a*)** Control, **(*b*)** OGD, **(*c*)** OGD + **(*d*)** OGD + NO-NBP M1 CM, **(*e*)** OGD + H_2_S-NBP M1 CM, **(*f*)** OGD + NOSH-NBP M1 CM groups. **(B)** A representative image of neuronal apoptosis. **(C)** Quantitative analysis of neuronal apoptosis (*n* = 3). **(D)** Quantitative analysis of cell viability percentage (*n* = 6). **(E)** Quantitative analysis of LDH release percentage (*n* = 6). Data are mean ± SD and were analyzed by one-way ANOVA followed by *post hoc* Tukey test: *^∗∗∗^P <* 0.001, *^∗∗^P* < 0.01, *^∗^P* < 0.05.

### Effects of Microglia Polarization on Post-OGD EC Survival and Integrity, and Impacts of NO-NBP, H_2_S-NBP, and NOSH-NBP-Treated M1 Microglial Conditioned Media on Post-OGD EC Survival

Although it is well-accepted that ischemia-induced over-activation of microglia damage the BBB, there are few reports assessing the role of microglia polarization in BBB viability and integrity. Therefore, different microglia CMs were applied to non-OGD or post-OGD ECs, which are the major BBB components. No variations were observed in cell viability, LDH release, TEER value and even the expression levels of ZO-1 and occludin in non-OGD ECs exposed to different microglia CMs (**Figures 8A–E**). Microglia polarization differently modulated post-OGD EC viability and integrity. M1-polarized CM aggravated OGD-caused EC damage, manifested by increased LDH release, and decreased cell viability, TEER and the expression levels of ZO-1 and occludin. In contrast, M2-polarized CM reversed these abnormalities in post-OGD ECs. The effects of CMs from NO-NBP, H_2_S-NBP, or NOSH-NBP-treated M1 microglia on post-OGD ECs were also investigated. NO-NBP, H_2_S-NBP, and NOSH-NBP tended to prevent M1 CM-induced death of post-OGD ECs, but only NOSH-NBP exhibited significant differences in cell viability and LDH release (*P* < 0.01 and *P* < 0.05 respectively, **Figures 8F,G**). Obviously, NOSH-NBP was the most effective.

**FIGURE 8:** **Effect of microglia polarization on post-OGD b.End3 endothelial cells (ECs) survival and function, and the effect of NO-NBP, H_2_S-NBP, or NOSH-NBP-treated M1 microglial condition media on post-OGD ECs survival.** BV_2_ microglia were treated with LPS (100 ng/mL) + IFN-γ (20 ng/mL), IL-4 (20 ng/mL), NO-NBP (10 μM), H_2_S-NBP (10 μM), NOSH-NBP (10 μM) or a combination of these agents for 24 h, followed by medium collection. After 3 h OGD, ECs were incubated with different condition media of microglia (M0, M1, M2, NO-NBP-M1, H_2_S-NBP-M1, or NOSH-NBP-M1), respectively. **(A)** Quantitative analysis of cell viability percentage (*n* = 6). **(B)** Quantitative analysis of LDH release percentage (*n* = 6). **(C)** Data of TEER assay. **(D)** Representative Western blot membranes for occludin and ZO-1 proteins expressions. **(E)** Quantitative analysis of occludin and ZO-1 proteins expressions (*n* = 3). **(F)** Quantitative analysis of cell viability percentage (*n* = 6). **(G)** Quantitative analysis of LDH release percentage (*n* = 6). Data are expressed as the mean ± SD and were analyzed by one-way ANOVA followed by *post hoc* Tukey test: *^∗∗∗^P <* 0.001, *^∗∗^P* < 0.01, *^∗^P* < 0.05.

### NOSH-NBP Downregulates Pro-inflammatory Cytokines Involved in the TLR4/MyD88/NF-κB Pathway and NLRP3 Inflammasome

The above results indicated that NOSH-NBP had great inhibitory effects on microglial inflammatory activation. We next explored the possible underlying mechanisms, whether the TLR4/MyD88/NF-κB pathway and NLRP3 inflammasome were involved. In ischemic stroke, the TLR4/MyD88/NF-κB pathway plays an important role in the expression of many proinflammatory mediators; meanwhile, maturity and secretion of proinflammatory mediators (IL-1β and IL-18) depend on NLRP3 inflammasome activation. *In vivo* data showed that NOSH-NBP (0.4, 0.2, and 0.1 mg/kg) alleviated tMCAO-induced over-expression of TLR4, MyD88, and p65 phosphorylation (**Figures 9A,B**). Meanwhile, NOSH-NBP (0.4, 0.2, and 0.1 mg/kg) inhibited NLRP3 inflammasome activation by decreasing NLRP3 and cleaved caspase-1 levels in the ischemic brain (**Figures 9A,C**). The release of pro-inflammatory mediators (IL-1β, IL-18, IL-6, and TNF-α) in the brain parenchyma was subsequently suppressed by NOSH-NBP (0.4, 0.2, and 0.1 mg/kg) (**Figure 9D**).

**FIGURE 9:** **NOSH-NBP suppresses the relative expression of M1-markers through the TLR4/MyD88/NF-κB pathway and NLRP3 inflammasome *in vivo* and *in vitro*.** *In vivo*, the model group and NOSH-NBP-treated group underwent tMCAO; the sham group underwent the same surgical procedure without the filament insertion. After MCAO being performed, mice in test compound groups were administrated with NOSH-NBP (0.4, 0.2, and 0.1 mm/kg) for 3 days. *In vitro*, BV_2_ microglia were treated with LPS (100 ng/mL) + IFN-γ (20 ng/mL), IL-4 (20 ng/mL), control siRNA, TLR4 siRNA, NOSH-NBP (10 μM) or a combination of these treatments. **(A)** Representative Western blot membranes for TLR4, MyD88, cytoplasm NF-κB, nucleus NF-κB, NLRP3 and caspase-1. **(B,C)** Quantitative analysis of TLR4, MyD88, cytoplasm NF-κB, nucleus NF-κB, NLRP3 and caspase-1 proteins expression levels (*n* = 3). **(D)** Quantitative analysis of pro-inflammatorty cytokines (IL-1β, IL-18, IL-6, and TNF-α) concentration (*n* = 5). **(E)** Representative Western blot membranes for TLR4, MyD88, cytoplasm NF-κB, nucleus NF-κB, NLRP3, and caspase-1. **(F,G)** Quantitative analysis of TLR4, MyD88, cytoplasm NF-κB, nucleus NF-κB, NLRP3, and caspase-1 protein expression levels (*n* = 3). **(H)** Quantitative analysis of pro-inflammatorty cytokines (IL-1β, IL-18, IL-6, and TNF-α) concentration (*n* = 5). **(I)** Representative western blot membranes for TLR4, MyD88, cytoplasm NF-κB, nucleus NF-κB, NLRP3, and caspase-1. **(J,K)** Quantitative analysis of TLR4, MyD88, cytoplasm NF-κB, nucleus NF-κB, NLRP3, and caspase-1 protein expression levels (*n* = 3). **(L)** Quantitative analysis of pro-inflammatorty cytokines (IL-1β, IL-18, IL-6, and TNF-α) concentration (*n* = 5). Data are expressed as the mean ± SD and were analyzed by one-way ANOVA followed by *post hoc* Tukey test: *^∗∗∗^P <* 0.001, *^∗∗^P* < 0.01, *^∗^P* < 0.05.

The effect of NOSH-NBP on the TLR4/MyD88/NF-κB pathway and NLRP3 inflammasome were further confirmed *in vitro*. Microglia are the major inflammatory cells of the CNS, and main cellular source of NLRP3 inflammasome in the brain. LPS+IFNγ-stimulated microglia produced large amounts of pro-inflammatory cytokines (IL-1β, IL-18, IL-6, and TNF-α), accompanied by TLR4/MyD88/NF-κB pathway and NLRP3 inflammasome activation. NOSH-NBP (10 μM) and IL-4 (20 ng/ml) significantly suppressed the high levels of pro-inflammatory mediators (IL-1β, IL-18, IL-6, and TNF-α) by inhibiting the TLR4/MyD88/NF-κB pathway activation and NLRP3 inflammasome; indeed, NOSH-NBP (10 μM) and IL-4 (20 ng/ml) treatment reduced the expression levels of TLR4, MyD88, and nuclear NF-κB, and decreased the expression levels of NLRP3 and caspase-1, respectively (**Figures 9E–H**). Moreover, blockade of TLR4 expression using siRNA significantly inhibited NF-κB, NLRP3 and caspase-1 expression levels, while combination of TLR4 siRNA and NOSH-NBP (10 μM) slightly altered the effects of TLR4 siRNA with no statistical significance (NS, *P* > 0.05; **Figures 9I–L**). These findings suggested that the TLR4/MyD88/NF-κB pathway and NLRP3 inflammasome were involved in the NOSH-NBP-modulatory effects on inflammatory response in ischemic stroke.

### NOSH-NBP Upregulates the Expression of M2 Markers by Enhancing PPARγ Nuclear Translocation

Peroxisome proliferator activated receptor gamma activation is positively related to M2 marker expression. To explore whether PPARγ plays a role in the regulatory mechanism of M2 polarization after NOSH-NBP treatment, PPARγ levels were assessed in tMCAO-treated mice and LPS-treated microglia by Western blot. As shown in **Figures 10A–D**, PPARγ expression was significantly increased in the nucleus but reduced in the cytoplasm in the tMCAO-NOSH-NBP and LPS+IFN-NOSH-NBP groups compared with the MCAO-and LPS+IFNγ-vehicle groups, respectively. Furthermore, the PPARγ inhibitor GM9662 remarkably altered the effects of NOSH-NBP on microglial M2 polarization, as reflected by decreased levels of M2-related markers (CD206, Ym1/2, and Arg1) with combined treatment of GM9662 and NOSH-NBP (**Figure 10E**).

**FIGURE 10:** **NOSH-NBP upregulates M2 markers by stimulating the nuclear translocation of PPARγ *in vivo* and *in vitro*.** *In vivo*, the model- group and NOSH-NBP-treated groups underwent tMCAO; the sham group underwent the same surgical procedure without the filament insertion. After MCAO completion, mice in the teat compound groups were administered with NOSH-NBP (0.4, 0.2, and 0.1 mm/kg) for 3 days. *In vitro*, BV_2_ microglia were treated with LPS (100 ng/mL) + IFN-γ (20 ng/mL), IL-4 (20 ng/mL), NOSH-NBP (10 μM), GM9662 (20 μM) or a combination of these treatments. **(A)** Representative Western blot membranes for cytoplasm PPARγ and nucleus PPARγ. **(B)** Quantitative analysis of cytoplasm PPARγ and nucleus PPARγ protein expression levels (*n* = 3). **(C)** Representative Western blot membranes for cytoplasm PPARγ and nucleus PPARγ. **(D)** Quantitative analysis of cytoplasm PPARγ and nucleus PPARγ protein expression levels (*n* = 3). **(E)** Quantitative analysis of mRNA expression levels of M2 markers: CD206, Ym1/2, and Arg1 (*n* = 6). Data are expressed as the mean ± SD and were analyzed by one-way ANOVA followed by *post hoc* Tukey test: ^∗∗∗^*P* < 0.001, ^∗∗^*P* < 0.01, ^∗^*P* < 0.05.

## Discussion

Ischemic stroke is a severe disease that causes great damage to human health, with limited effective treatment available. Increasing evidence demonstrates that NO and H_2_S have critical roles in ischemic brain injury (Zhou et al., 2012). NOSH-NBP, a novel double-donor, is capable of releasing both NO and H_2_S at a moderate levels. Our previous results showed that preventive administration of NOSH-NBP could decrease infarct volume, brain edema, and neurological deficit scores, and alleviate oxidative stress in tMCAO-treated rats (Yin et al., 2016). Therefore, as a potential agent, NOSH-NBP is worth paying more attention to, revealing its therapeutic effects and underlying mechanisms in ischemic stroke.

In ischemic stroke, endogenous NO is synthesized by nitric oxide synthases (NOSs), which include three isoforms, i.e., inducible (nNOS and iNOS) and endothelial (eNOS). Different from NO produced by nNOS and iNOS, eNOS-derived NO is beneficial for stroke (Samdani et al., 1997). Endogenous H_2_S in the brain is produced by three enzymes, namely cystathionine β-synthase (CBS), cystathionine γ-lyase (CSE), and the tandem enzymes cysteine aminotransferase (CAT) and 3-mercaptopyruvate sulfurtransferase (3-MST). Absence of CSE or CAT/3-MST aggravates ischemic brain injury (Zheng et al., 2015). Many preclinical studies revealed that exogenous NO donors (e.g., SNP, sydnonomines, NONOates, and NO-NBP) and H_2_S donors (e.g., NaSH, ADTOH, and H_2_S-NBP) are beneficial in ischemic stroke (Willmot et al., 2005; Zhuang et al., 2010; Wang X. et al., 2014; Wang Y. et al., 2014). In this study, we firstly performed both *in vivo* and *in vitro* experiments to explore whether NOSH-NBP, in comparison with the single-donors, i.e., NO-NBP and H_2_S-NBP, have therapeutic effects on ischemic stroke. As shown above, therapeutic treatment with NOSH-NBP time-dependently decreased neurological deficit and infarct volume, and was more potent than NO-NBP and/or H_2_S-NBP. To confirm the role of NO or H_2_S in NOSH-NBP effects in ischemic stroke, we selectively eliminated NO or H_2_S in NOSH-NBP with NO and H_2_S scavengers, namely Carboxy-PTIO and BSS respectively, both of which greatly weakened the anti-ischemia effects of NOSH-NBP.

Historically, the fundamental premise of neuroprotection simply focuses on preventing neuronal death in stroke. However, despite tremendous advances have been achieved in the molecular biology of intra-neuronal mechanisms and pathways, multiple exploratory trials for neuroprotection have failed, and a clinically effective neuro-protectant does not exist (del Zoppo, 2006). The failure of neuro-protectants led to a shift in perspective from focusing on the neuron alone to paying attention to the complexity of neuron-supplying microvessels, and supportive cells (glial cell, and resident inflammatory cell), all of which are included in the NVU concept (Guo and Lo, 2009). Apart from having direct effects on cells, ischemia also initiates inflammation, increases microvascular permeability (which causes brain edema), and induces local hemorrhage. Ischemic stroke has such effects as it is actually a cerebrovascular disorder affecting neuronal function. Neurons and microvessels respond equally rapidly to cerebral ischemic insults. As a powerful vasodilator, vascular-derived NO can modulate the blood flow. NO also has an antiplatelet effect and can inhibit leukocyte adhesion/migration to the endothelium, which is beneficial for microvessels (Willmot et al., 2005). Also, H_2_S treatment potentially protects BBB integrity and function in some CNS diseases, such as cerebral ischemia and Alzheimer (Kamat et al., 2016). The present study demonstrated that therapeutic administration of NOSH-NBP not only prevented neuronal death, but also alleviated neurovascular damage in the penumbral region. NOSH-NBP decreased BBB permeability and brain edema. In addition, ischemia-caused loss of barrier function permeability involves dysfunction of the tight junction proteins occludin and ZO-1, an effect improved by NOSH-NBP treatment. Furthermore, glial activation/transformation is another important feature in NVU dysfunction. Moreover, we provided evidence that NOSH-NBP can suppress microglial activation and modulate microglial polarization, contributing to the beneficial effects of NOSH-NBP on tMCAO-treated mice.

Microglia are the major immune cells in the CNS (Bushnell, 2008). Additionally, peripheral macrophages infiltrate into the CNS after tMCAO from hours to days, a bridge between the CNS and periphery immune system. Recently, it was found that activated microglia/macrophages act as double-edged swords, depending on phenotypes. For instance, the M1 phenotype accelerates neuronal death and inflammation by generating a number of pro-inflammatory mediators (CCL3, IL-β, and TNFα), while the M2 phenotype improves neuronal survival and tissue repair by producing anti-inflammatory mediators (CD206, Ym1/2, and Arg1) (Hu et al., 2012). The above *in vivo* results indicated that NOSH-NBP reduced the levels of M1 pro-inflammatory mediators, and increased those of M2 anti-inflammatory mediators. To confirm the modulatory effects of NOSH-NBP on microglia/macrophage polarization *in vitro*, BV_2_ microglia/BMDM were treated with OGD, LPS + IFNγ and IL-4, respectively. In line with *in vivo* results, NOSH-NBP inhibited M1 polarization and promoted M2 polarization in BV_2_ microglia/BMDM, as reflected by changes in mRNA levels of M1/M2-related genes. As mentioned above, NO and H_2_S are important modulators of inflammation. Therefore, we assessed the roles of NO and H_2_S in the microglia modulatory effects of NOSH-NBP. NO and H_2_S-donor groups both contributed to the inhibitory effects of NOSH-NBP on M1 polarization, as Carboxy-PTIO and BSS both greatly weakened NOSH-NBP effects on M1-related mRNA. However, only BSS blunted the effect of NOSH-NBP on M2-related gene expression, suggesting that H_2_S-donor group not NO-donor group is involved in NOSH-NBP induced M2 polarization. From a physiological perspective, although NO and H_2_S have some similar functions, such as blood vessel relaxation, they act on different downstream targets, including respectively soluble guanylyl cyclase/cyclic guanosine monophosphate (sGC-cGMP) and the potassium (K^+^) channel (Mustafa et al., 2009). In peripheral macrophages, the expression of CD206, a M2 marker, is insensitive to the change of endogenous NO content, whereas elevation of H_2_S production by CBS overexpression not only inhibits M1 markers but also promotes M2 markers (Chao et al., 2015; Kalish et al., 2015). These observations provide the possible differences between NO and H_2_S in the regulation of microglial polarization.

Promoting M2 polarization of microglia is very significant in neuroprotection (Hu et al., 2012). To emphasize the significance of NOSH-NBP’s modulatory effects on microglia polarization, we performed a CM experiment in BV_2_ microglia and primary neurons. Consistent with previous research, M1 microglia CM aggravated post-OGD death of primary neurons. Importantly, post-OGD primary neurons treated with the CM from NOSH-NBP-pretreated M1 microglia had a higher survival rate compared with those treated with M1 microglia CM only, indicating that NOSH-NBP neuroprotection against ischemic stroke injury is at least partially attributed to its promotion of M1–M2 switch.

Increasing evidence suggests that activated microglia modulate tight junction genes, which are critical to BBB integrity and function (Sumi et al., 2010). Moreover, microglia tend to migrate from ischemic to perivascular areas in MCAO-treated animals, implying that ischemia strengthens their contact (Li et al., 2016). Yet, few reports have assessed the role of different microglial phenotypes in BBB function after ischemia. For clarification, we performed CM experiments in BV_2_ microglia and ECs. Interestingly, no-OGD ECs treated with CM from M0, M1, and M2 microglial phenotypes, respectively, caused no changes of EC survival, TEER value, and the tight junction-associated proteins occludin and ZO-1. CM from M1 and M2 microglia differently modulated post-OGD EC viability and integrity; CM from M1 microglia aggravated post-OGD EC injury, while those from M2 microglia alleviated post-OGD EC injury, as reflected by changes of ECs viability, TEER value, and occludin and ZO-1 expression levels. This finding supports that the notion of M1–M2 switch not only exhibits neuroprotection but also neurovascular protection. Therefore, it can be inferred that polarization of microglia from M1 toward M2 is beneficial for NVU integrity and function in ischemic stroke. Meanwhile, our data confirmed that the modulatory effects of NOSH-NBP on microglial polarization contributes to its neurovascular protection, as indicated by increased EC survival after treatment with CM from NOSH-NBP-pretreated M1 microglia compared with treatment with M1 microglia CM only.

We also attempted to explore the regulatory mechanisms of NOSH-NBP effects on microglial polarization, which involve some signaling pathways. The TLR4/MyD88/NF-κB pathway is essential for microglial activation for toxicity in ischemic stroke (Wang et al., 2015). Activation of TLR4-MyD88 leads to the subsequent activation of NF-κB, which triggers the transcription of pro-inflammatory cytokines, such as IL-1β, IL-6, and TNF-α (Shao et al., 2016). As shown above, NOSH-NBP inhibited the TLR4/MyD88/NF-κB pathway by suppressing TLR4 and MyD88 expression levels, as well as p65 phosphorylation, *in vivo* and *in vitro*. Moreover, production and secretion of pro-inflammatory cytokines require inflammasome activation. As a M1-related marker, the NLRP3 inflammasome, composed of NLRP3, apoptosis-associated speck-like protein containing a caspase recruitment domain (ASC) and caspase-1, also has a critical role in M1 microglial activation (Girard et al., 2013; Yang et al., 2014). It has been demonstrated that NF-κB is also involved in NLRP3 inflammation activation by inducing NLRP3 transcription (Bauernfeind et al., 2009). Our results verified that NOSH-NBP inhibits the NLRP3 inflammasome *in vivo* and *in vitro*. Experiments involving TLR4 knockdown using the siRNA technology in microglia were performed to further elucidate the inhibitory effects of NOSH-NBP on the TLR4/MyD88/NF-κB pathway and NLRP3 inflammasome, were responsible for its inhibitory effects on M1 microglia activation. PPARγ, as a nuclear transcriptional factor, is highly expressed in many immune cells, e.g., microglia and macrophages. Its activation plays a protective role in the CNS, and increases M2-marker levels in microglia/macrophages and tMCAO-treated mice, e.g., Arg-1 and CD206 (Sundararajan et al., 2006; Pan et al., 2015). In this study, NOSH-NBP enhanced PPARγ activation by increasing its nuclear translocation of PPARγ, promoting NOSH-NBP effects on M2 polarization. Moreover, these findings were further confirmed by the use of PPARγ antagonist GW9662 that significantly altered NOSH-NBP effects on M2-markers.

We previously demonstrated that NOSH-NBP could release both moderate amounts of NO (0.1 mM NOSH-NBP approximately releases 10.57 μM NO) and H_2_S (about 4.4% conversion of NOSH-NBP to H_2_S) *in vitro*; however, the releasing rate, time, and position of NO and H_2_S in NOSH-NBP after administration *in vivo* need to be confirmed. Additionally, neuroinflammation is a hallmark of various neurodegenerative diseases, such as Alzheimer’s disease (AD), Parkinson’s disease (PD), and multiple system atrophy (MSA), and is mainly mediated by microglia in the brain (Merazríos et al., 2016). Recently, it was suggested that switching of M1/M2 phenotypes could constitute a new therapeutic tool for preventing brain injury from neurodegenerative diseases (Tang and Le, 2016). Considering the favorable regulation of NOSH-NBP on microglia polarization, further study to assess its effects on neurodegenerative diseases is warranted.

In summary, this study demonstrated that: (1) NOSH-NBP has potent therapeutic effects on ischemic stroke in mice by inhibiting neuronal death, ameliorating BBB impairment and promoting microglial M1–M2 phenotype switch, providing superior effects compared with NO-NBP and/or H_2_S-NBP; (2) NO and H_2_S-donor groups contribute to the anti-ischemic effects of NOSH-NBP, including neuroprotection, neurovascular protection, and reduced microglial M1 polarization, with only the H_2_S-donor group involved in promoting microglial M2 polarization; (3) NOSH-NBP exhibits protective effects on post-OGD neurons and ECs by modulating microglial polarization; (4) NOSH-NBP inhibits M1-like microglial activation by regulating the TLR4/MyD88/NF-κB pathway and NLRP3 inflammasome, and promotes M2-like microglial activation by enhancing the nuclear translocation of PPARγ. These findings suggest that NOSH-NBP may constitute a new tool for treating ischemic stroke.

## Author Contributions

JJ designed the study and drafted the manuscript. PX analyzed the data. JJ, PX, TL, LL, XX, GL, and YZ carried out the experiments. All authors contributed to this study and have approved the final manuscript.

## Conflict of Interest Statement

The authors declare that the research was conducted in the absence of any commercial or financial relationships that could be construed as a potential conflict of interest.

## Abbreviations

ADTOH: 5-(4-hydroxyphenyl)-3H-1,2-dithiole-3-thione
Arg1: arginase 1
BBB: blood–brain barrier
BSS: bismuth (III) subsalicylate
CCL3: chemokine (CC motif) ligand 3
EB: Evans blue
ELISA: enzyme-linked immunosorbent assay
4-HBN: 4-hydroxybutyl nitrate
H_2_S: hydrogen sulfide
IL: interleukin
LDH: lactate dehydrogenase
LPS: lipopolysaccharide
MyD88: myeloid differentiation factor 88
NBP: 3-*n*-butylphthalide
NF-κB: nuclear factor kappa B
NLRP3: NOD-like receptor 3
NO: nitric oxide
NVU: neurovascular unit
OGD: oxygen-glucose deprivation
PPARγ: peroxisome proliferator activated receptor gamma
TEER: trans*-*endothelial electrical resistance
TLR4: toll-like receptor 4
tMCAO: transient middle cerebral artery occlusion
TNF-α: tumor necrosis factor
TTC: 2, 3, 5-triphenyltetrazolium chloride
ZO-1: zonula occluden-1.
